# AR-v7 protein expression is regulated by protein kinase and phosphatase

This article has been retracted.

**DOI:** 10.18632/oncotarget.5608

**Published:** 2015-09-10

**Authors:** Yinan Li, Ning Xie, Martin E. Gleave, Paul S. Rennie, Xuesen Dong

**Affiliations:** ^1^ Vancouver Prostate Centre, Department of Urologic Sciences, University of British Columbia, Vancouver, Canada

**Keywords:** castration resistant prostate cancer, AR-v7, serine phosphorylation, protein stability, PP-1 and Akt

## Abstract

Failure of androgen-targeted therapy and progression of castration-resistant prostate cancer (CRPC) are often attributed to sustained expression of the androgen receptor (AR) and its major splice variant, AR-v7. Although the new generation of anti-androgens such as enzalutamide effectively inhibits AR activity, accumulating pre-clinical and clinical evidence indicates that AR-v7 remains constitutively active in driving CRPC progression. However, molecular mechanisms which control AR-v7 protein expression remain unclear. We apply multiple prostate cancer cell models to demonstrate that enzalutamide induces differential activation of protein phosphatase-1 (PP-1) and Akt kinase depending on the gene context of cancer cells. The balance between PP-1 and Akt activation governs AR phosphorylation status and activation of the Mdm2 ubiquitin ligase. Mdm2 recognizes phosphorylated serine 213 of AR-v7, and induces AR-v7 ubiquitination and protein degradation. These findings highlight the decisive roles of PP-1 and Akt for AR-v7 protein expression and activities when AR is functionally blocked.

## INTRODUCTION

Androgen-targeted therapy (ATT) is the primary treatment for metastatic prostate cancers. It either blocks androgen synthesis or prevents the androgen receptor (AR) from being transcriptionally active. Unfortunately, tumors eventually progress into incurable castration-resistant prostate cancer (CRPC) and are most often driven by re-activated AR signaling via mechanisms involving AR gene amplification, gain-of-function mutations and intratumoral steroidogenesis [1–3]. While the new generation of anti-androgens such as enzalutamide (ENZ) targets the ligand binding domain (LBD) of the AR and blocks AR activity efficiently, resistance to ENZ develops in essentially all patients [4, 5]. Emerging pre-clinical and clinical evidence supports the idea that cancer cells can utilize RNA splicing mechanisms to generate AR variants and escape from ATT [6–10]. Among several AR splice variants, AR-v7 is the most highly expressed in prostate tumors. Lacking the LBD, AR-v7 is constitutively active and can drive tumor progression even under ENZ treatment [6, 11]. Understanding the molecular mechanisms which control AR-v7 protein expression is therefore important to develop new therapies for CRPC.

Generation of AR-v7 mRNA is through an alternative RNA splicing process, which is coupled with AR gene transcription, enhanced by castration conditions, and facilitated by AR gene amplification/rearrangement [12, 13]. However, AR-v7 protein has to be stabilized in cells in order to exert its functions. No mechanistic study on the regulation of AR-v7 protein expression has been performed. Previous studies have shown that post-translational modifications of full length AR (AR-FL), such as phosphorylation modification at multiple serine residuals, regulate not only AR-FL protein stability but also AR-FL subcellular localization and transcriptional activity [14]. Akt protein kinase phosphorylates serine 213 and 791 of AR-FL, activates Mdm2 ubiquitin ligase and induces AR-FL protein degradation by proteasome pathway [15, 16]. Protein phosphatase-1 (PP-1) was demonstrated to de-phosphorylate only serine 650 and increase AR protein expression and activity [17]. AR-v7 does not have serine 650 and 791. Whether PP-1 and Akt regulate AR-v7 phosphorylation and protein degradation remains unknown.

Genetic heterogeneity of prostate cancer cells is a significant challenge for cancer therapy and may produce profound impacts on AR-v7 protein expression. For example, cells carrying AR gene amplification or rearrangement express high levels of AR-v7 mRNAs to be translated [12, 13]. Cells with loss-of-function of PTEN also become resistant to castration-induced apoptosis due to overactive Akt signaling [18, 19]. However, inhibitors for PI3K/Akt signaling may also increase AR protein expression through feedback loop mechanisms [18]. The consequence of these intratumoral mutations is that not all cells within a tumor would respond equally to the inhibitors for AR and PI3K/Akt signaling. Dissecting the genetic variations in association with AR-v7 protein expression is therefore important to direct therapy strategy for CRPC.

In this study, we apply multiple prostate cancer lines with different genetic backgrounds to study differential activation of PP-1 and Akt by AR inhibition. Activated PP-1 and Akt in turn determine the extent of serine 213 phosphorylation, pSer(213), of AR-v7 and Mdm2-mediated AR-v7 protein degradation. These results link genetic backgrounds of prostate cancer cells with AR-v7 protein stability when cancer cells are under AR inhibition conditions.

## RESULTS

### Differential activation of PP-1 and Akt by AR inhibition determines AR and AR-v7 protein expression

We chose LNCaP, LNCaP95, 22Rv1 and VCaP cells to study AR protein expression under castration conditions, because they have representative genetic aberrations in AR and PTEN genes in addition to many other mutations in their genome. LNCaP, 22Rv1 and VCaP cells were cultured in medium containing fetal bovine serum (FBS) and then switched to androgen deprived medium plus 5μM of ENZ for maximum androgen blockade (MAB) (Figure 1). LNCaP95 cells were routinely maintained in androgen deprived medium and were treated with ENZ. In all these cells, both endogenous mRNA levels of AR-FL and AR-v7 increased (Figure S1), which is consistent with the previous study that indicated androgen-activated AR inhibited AR gene transcription [20]. However, these cells responded to MAB differently in AR protein expression (Figure 1). MAB rapidly reduced AR-FL and AR-v7 protein levels, but increased pSer(213) of AR-FL and AR-v7 in PTEN-deficient LNCaP and LNCaP95 cells (Figure 1A). Reduced AR protein levels were correlated with increased levels of pAkt and phosphorylated Mdm2 (pMdm2), but decreased PP-1 protein levels. Since the pSer(213) antibody recognizes a non-specific band overlapping with AR-v7, increased pSer(213) levels of AR-v7 were therefore detected by immunoprecipitation with AR antibody followed by immunoblotting with pSer(213) antibody (Figure 1B). It should be noted that similar amounts of AR-FL and AR-v7 proteins were precipitated by the fixed amount of AR antibody used in these assays. However, the proportions of phosphorylated AR-FL and AR-v7 in the precipitated AR proteins were increased by MAB (Figure 1B). In PTEN-sufficient 22Rv1 cells, where undetectable pAkt were expressed, MAB increased AR-FL and AR-v7 but reduced AR pSer(213) protein levels (Figure 1A and 1B). Concurrently, PP-1 protein levels were increased, while pMdm2 levels were decreased (Figure 1A). However in PTEN-sufficient VCaP cells, MAB induced AR-FL and AR-v7 protein expression without alteration of pSer(213) levels. MAB had no effect on Akt, PP-1 and Mdm2 activation. Therefore, enhanced AR-FL and AR-v7 protein expression in VCaP cells (bearing AR gene amplification) by MAB was likely related to increased AR gene transcription (Figure S1).

**Figure 1:** Differential activation of PP-1 and Akt by ENZ determines AR and AR-v7 protein expression LNCaP, 22Rv1 and VCaP cells were cultured in medium containing 5% FBS and then treated with medium containing 5% charcoal stripped serum (CSS) and 5μM of enzalutamide (ENZ) for 0-24 hours. LNCaP95 (LN95) cells were maintained in medium containing 5% CSS and then treated with 5μM of enzalutamide (ENZ) for 0-24 hours. **A.** Whole cell lyses were extracted. AR-FL, AR-v7, phosphor-AR(ser213), phosphor-Akt(ser473), total Akt, total PP-1, phosphor-Mdm2(ser166), total Mdm2 and β-actin were measured by immunoblotting. **B.** Protein lysates from LNCaP95 and 22Rv1 cells were immunoprecipitated with AR (N-20) antibody. Associated proteins were immunoblotted with phosphor-AR(Ser213) and AR(N-20) antibodies. **C.** LNCaP95 cells transfected with control siRNA or pooled siRNA against Akt1 and Akt2. **D.** 22Rv1 cells were transfected with constitutive Akt (cAkt) or dominant negative Akt (dAkt) expression vector for 24 hours. Cells were treated with medium containing 5% CSS plus 5μM ENZ for 0-24 hours. AR-FL, AR-v7, phosphor-AR(ser213), phosphor-Akt(ser473), total Akt, total PP-1, phosphor-Mdm2(ser166), total Mdm2 and β-actin were detected by immunoblotting. Experiments were repeated more than three times and only one set of results was shown.

To determine whether PP-1 and Akt were causal factors determining protein expression of AR-FL and AR-v7, we first depleted Akt expression by siRNA in PTEN-deficient LNCaP95 cells (Figure 1C). Akt depletion resulted in increased AR-FL and AR-v7 protein levels under MAB. Concurrently, MAB increased PP-1 and reduced the extent of Mdm2 phosphorylation when compared with control siRNA transfected cells. Next, constitutively active Akt (cAkt) was introduced into PTEN-sufficient 22Rv1 cells. AR-FL, AR-v7 and PP-1 protein levels were significantly reduced by MAB, while AR pSer(213) and pMdm2 levels were upregulated when compared with 22Rv1 cells transfected with dominant negative Akt (dAkt) (Figure 1D). Together, these results show that MAB differentially activates PP-1 and Akt signaling in prostate cancer cells, thereby determining AR-FL and AR-v7 protein expression.

### PP-1 regulates AR-FL and AR-v7 protein degradation through proteasome pathway

PP-1 was demonstrated to de-phosphorylate only serine 650 in AR LBD and regulate AR-FL protein stability [17]. In this study, we showed that PP-1 specific inhibitor, tautomycetin (TMC), reduced both AR-FL and AR-v7 protein expression but increased AR pSer(213) levels in both time- and dose-dependent manners in LNCaP, LNCaP95 and 22Rv1 cells (Figure 2A and S2A). Overexpression of PP-1 catalytic isoforms (PP-1α, PP-1β and PP-1γ), but not mutant PP-1 with destroyed enzymatic activity, enhanced AR-FL and AR-v7 protein levels (Figure 2B and 2C). Concurrently, pSer(213) levels of AR were decreased. When cells were treated with cycloheximide (CHX), AR-FL and AR-v7 protein degradation rates were accelerated by TMC in a time-dependent manner (Figure 2D, Figure S2B-C). By contrast, proteasome inhibitors epoxomicin and MG132 prevented TMC from inducing AR protein degradation (Figure 2E).

**Figure 2:** PP-1 regulates AR-FL and AR-v7 protein degradation through proteasome pathway **A.** LNCaP95 (LN95), LNCaP and 22Rv1 cells were treated with 5μM of tautomycetin (TMC) for 0-24 hours. **B.** LNCaP95, 22Rv1 and 293T cells were transfected with expression vector for control, HA-tagged PP-1α, β or γ. **C.** LNCaP95, 22Rv1 and 293T cells were transfected with plasmid encoding control, HA-tagged PP-1γ or PP-1γ mutant (H125A). 293T cells were also transfected with AR-FL and AR-v7 expression vector (B and C). AR-FL, AR-v7, phosphor-AR(ser213), HA-tagged PP-1 and β-actin were detected by immunoblotting. **D.** LNCaP95 cells were treated with 50μg/ml of cycloheximide (CHX) plus either vehicle or 5μM of TMC for 0-24 hours. AR-FL and AR-v7 were detected by Western blotting. Densitometry analyses of AR-FL and AR-v7 levels were normalized to β-actin. Results were from triplicate experiments. **E.** LNCaP95, PC3(AR-FL), PC3(AR-v7) and LNCaP cells were treated with 0, 2 and 5μM of TMC plus vehicle, 100nM of epoxomicin (EPOX) or 2μg/ml of MG132 for 24 hours. AR-FL and AR-v7 proteins were detected by Western blotting. Experiments were repeated more than three times and only one set of results was shown.

Gain- and loss-of-function of PP-1 did not alter AR gene transcription (Figure S3A-D) as well as AR-FL and AR-v7 RNA splicing processes (Figure S3E-H). We further showed that upregulation of AR-FL and AR-v7 protein expression by PP-1 also enhanced their transcriptional activities (Figure S4A-F). By contrast, RNA silencing of PP-1 reduced transcription of endogenous AR targeted genes (Figure S4G and S4H). Together, these results indicate that PP-1 regulates AR-FL and AR-v7 protein degradation through the proteasome pathway. Independent to Akt activity, this PP-1 function is active in both PTEN-sufficient 22Rv1 and 293T cells and PTEN-deficient LNCaP, LNCaP95 and PC3 cells.

### PP-1 regulates AR-FL and AR-v7 protein stability through Mdm2 ubiquitin ligase

Both PP-1 and Akt were reported to regulate Mdm2 phosphorylation, thus its E3 ligase activity [21, 22]. To determine whether PP-1 regulated AR-FL and AR-v7 protein stability through Mdm2, we first showed that pMdm2 levels were increased, while total Mdm2 levels remained unchanged in LNCaP95 and 22Rv1 cells treated with TMC or PP-1 siRNA (Figure 3A and 3B). These results also indicated that PP-1 regulation of AR protein expression was independent to Akt activation, because minimal Akt activation existed in 22Rv1 cells (Figure 3B). By contrast, overexpression of PP-1 but not PP-1 mutant reduced pMdm2 levels (Figure 3C). When Mdm2 expression was depleted by siRNA, TMC cannot reduce AR-FL and AR-v7 protein levels (Figure 3D). Additionally, Mdm2 overexpression reduced the function of PP-1 in upregulating AR-FL and AR-v7 protein expression (Figure 3E). Furthermore, Mdm2 enhanced AR-v7 (Figure 3F) and AR-FL (Figure 3G) ubiquitination. Overexpression of PP-1 decreased, while TMC or cAkt increased AR-v7 and AR-FL ubiquitination in both PTEN-sufficient 293T cells and PTEN-deficient PC3 cells (Figure S5). These results demonstrated that Mdm2 mediated PP-1 actions in controlling AR-FL and AR-v7 protein stability.

**Figure 3:** PP-1 regulates AR-FL and AR-v7 protein stability through Mdm2 ubiquitin ligase LNCaP95 (LN95) and 22Rv1 cells were: **A.** treated with 0-5μM of TMC for 24 hours or **B.** transfected with control or pooled PP-1α/β/γ siRNA for 48 hours or **C.** transfected with plasmid encoding control, PP-1γ or PP-1γ mutant (H125A) for 24 hours. AR-FL, AR-v7, phosphor-Mdm2(ser166), total Mdm2, phosphor-Akt(ser473), PP-1 and Akt proteins (only PP-1α was shown) were detected by immunoblotting. **D.** LNCaP95 and 293T(AR-v7) cells were transfected with control or Mdm2 siRNA and then treated with either vehicle or 5μM of TMC for 48 hours. AR-FL, AR-v7, Mdm2 and β-actin were detected by immunoblotting. **E.** 293T cells were co-transfected with AR-FL and AR-v7 expression vector. Cells were also transfected with control or Mdm2 plasmid in addition to control, PP-1γ or PP-1γ mutant (H125A) plasmid as indicated for 24 hours. AR-FL, AR-v7, PP-1γ and β-actin were detected by immunoblotting. 293T cell were transfected with AR-v7 **F.** or AR-FL **G.** expression vector. Cells were also transfected with ubiquitin vector plus either control or Mdm2 plasmid, and then treated with 2μg/ml of MG132 for 16 hours. *In vivo* ubiquitination assays were performed as described in the *Material and Method* section. All experiments (A-G) were repeated at least three times with one set of results shown in the figure.

Although our results showed that AR-FL and AR-v7 proteins were regulated similarly by PP-1 and Akt activities, we focused on AR-v7, the major AR splice variant in CRPC tumors in the current study. Ligand-dependent transactivation of AR-FL is potently suppressed by MAB regardless of AR-FL protein expression. However, AR-v7 is constitutively active and its protein expression could drive CRPC progression.

### AR-v7 ubiquitination results in AR-v7 localization to cytoplasm for protein degradation

We utilized LNCaP cells expressing GFP-tagged AR-v7 to study AR-v7 subcellular localization under differential activation of PP-1 and Akt. Fluorescence microscopy studies showed that TMC not only reduced AR-v7 protein levels, but also induced AR-v7 localization in cytoplasm (Figure 4A). These changes were associated with increased levels of pMdm2, which was mainly localized in nuclei. Similar observations were also obtained from 22Rv1 cells, in which cAkt was introduced in the cells (Figure 4B). Reduced AR-v7 protein levels were accompanied by AR-v7 localization in cytoplasm, concurrently with increased pMdm2 levels. These results suggested that Mdm2-mediated ubiquitination of AR-v7 was in nuclei, after which ubiquitinated AR-v7 was exported to cytoplasm for protein degradation. To test this hypothesis, we performed *in vivo* ubiquitination assays (Figure 4C–4E). Protein lyses from 293T cells expressing AR-v7 were first fractioned into nuclear and cytosol extracts in denature buffers to disrupt any non-covalent protein interactions. Following immunoprecipitation with AR antibody and immunoblotting with AR or ubiquitin antibody, AR-v7 ubiquitination was observed only in cytoplasm fraction. AR-v7 ubiquitination levels were decreased by PP-1, but increased by either TMC or cAkt. Similar results were also observed for the localization of ubiquitinated AR-FL (Figure S6).

**Figure 4:** AR-v7 ubiquitination results in AR-v7 localization to cytoplasm for protein degradation **A.** LNCaP cells were transfected with GFP-tagged AR-v7 plasmid and then treated with 5μM of TMC for 0, 2 or 4 hours. **B.** 22Rv1 cells were transfected with GFP-tagged AR-v7 plasmid together with either cAkt or dAkt expression vector for 24 hours. Cells were fixed, immunostained with phosphor-Mdm2(ser166) antibody, and examined by fluorescence microscope. 293T cells were transfected with AR-v7 plasmid (C and E). PC3 cells were stably introduced with exogenous AR-v7 protein **D.**. Cells were co-transfected with either control or PP-1 plasmid **C.**, or treated with vehicle or 5μM of TMC **D.** or transfected with dAkt or cAkt expression vector for 24 hours **E.**. Cells were also treated with 2μg/ml of MG132 for another 16 hours. Cytoplasmic and nuclear fractions of protein lysis were extracted. Histone 3 (H3) and tubulin were detected by immunoblotting and were used as markers to confirm the efficacy of cytosol and nuclear fraction. *In vivo* ubiquitination assays were performed as described in the *Material and Method* section. All experiments were repeated at least three times with one set of results shown in the figure.

### PP-1 and Akt regulate pSer(213) of AR-v7 and Mdm2-mediated AR-v7 ubiquitination

To investigate other potential serine phosphorylation sites targeted by PP-1 and Akt, we also performed site-directed mutagenesis to replace serine 213, 293, 424, 515 and 578 with alanine in AR-v7. Only AR-v7 (S213A) protein expression did not respond to gain- and loss-of-function of PP-1 (Figure 5A and 5B) or cAkt overexpression (Figure 5C). Co-immunoprecipitation assays indicated that AR-v7 (S213A) protein cannot be recognized by the antibody for pSer213 (Figure S7). Co-immunoprecipitation assays also showed that AR-v7 (S213A) did not form a protein complex with Mdm2 (Figure 5D). *In vivo* ubiquitination assays showed that TMC induced AR-v7 ubiquitination was significantly reduced (Figure 5E). Furthermore, AR-v7 (S213A) protein was resistant to TMC- or cAkt-induced protein degradation and remained in nuclei (Figure 5F and 5G). Together, these results demonstrate that PP-1 and Akt target pSer(213) in AR-v7 and regulate Mdm2-mediated AR-v7 protein stability.

**Figure 5:** PP-1 and Akt regulate pSer(213) of AR-v7 and Mdm2-mediated AR-v7 ubiquitination and protein degradation 293T cells were transfected with wild type or mutant AR-v7 expression vector. **A.** Cells were also transfected with control, PP-1γ, PP-1γ mutant (H125A) vector; **B.** cells were treated with either vehicle or 5μM of TMC; or **C.** cells were transfected with control, cAkt or dAkt expression vector for 24 hours. AR-v7, PP-1γ, Akt and β-actin were detected by immunoblotting. 293T cells were transfected with wild type or mutant AR-v7 expression vector. **D.** Immunoprecipitation assays were performed using either control IgG or Mdm2 antibody. Associated proteins were detected by AR or Mdm2 antibody. **E.** Cells were also treated with 2μg/ml of MG132 for another 16 hours. *In vivo* ubiquitination assays were performed as described in the *Material and Method* section. All experiments were repeated at least three times with one set of results shown in the figure. **F.** LNCaP cells were transfected with expression vector encoding flag-tagged wild type or mutant AR-v7 and then treated with 5μM of TMC for 0 or 4 hours. **G.** 22Rv1 cells were transfected with expression vectors encoding flag-tagged wild type and mutant AR-v7 plasmid. Cells were also transfected with either cAkt or dAkt plasmid for 24 hours. Cells were fixed, immunostained with Flag-tag antibody and examined by fluorescence microscope.

## DISCUSSION

Enhanced expression of AR splice variants had been demonstrated to be one of the key mechanisms contributing to CRPC [6–11, 23, 24]. AR variants can either form homodimer or heterodimer with AR-FL to resume AR signaling under castration conditions [25]. However, mechanisms controlling protein expression of AR variants remain unclear. In this study, we report several new findings: i) differential activation of PP-1 and Akt by MAB is determined by the genetic backgrounds of prostate cancer cells, and thereby controls AR-v7 protein stability; ii) PP-1 targets pSer(213) of AR-v7, prevents Mdm2 recruitment and Mdm2-mediated AR-v7 protein degradation by ubiquitin-proteasome pathway; and iii) Akt signaling regulates AR-v7 protein expression. While ongoing clinical trials test the efficacy of co-targeting AR and Akt signaling in CRPC, both treatments can increase AR-v7 protein expression. These results raise the concern that cancer cells may gain growth advantage once the AR-v7 protein level is upregulated and stabilized when both AR and PI3K/Akt signaling are both suppressed. Our findings therefore support the idea that targeting protein kinases or phosphatases may suppress AR-v7 expression and AR-v7 driven tumor growth.

Heterogeneity of prostate tumors is challenging, because ATT could effectively destroy many, but not all, cancer cells within tumors. Enrichment of cell populations carrying a variety of genetic mutations are frequently detected in CRPC [26]. Genome-wide profiling reports even broader ranges of genetic heterogeneity beyond mutations associated with protein components that are associated with AR and PI3K/Akt signaling [26]. PP-1 gene amplifications, as well as mutations in several PP-1 regulatory proteins, have been identified, implying that the PP-1 signaling is also aberrantly regulated at the genome level [26, 27]. In this study, our choice of only four prostate cancer cell lines presents readily distinct patterns of cellular responses to AR inhibition. AR-v7 is one among many other proteins, whose phosphorylation modification and protein expression is differentially regulated. Given the important role of AR-v7 for CRPC progression, our results emphasize that profiling AR-v7 protein expression, as well as genetic alterations associated with PP-1 and Akt signaling, may be required to direct treatments for individual cancer patients.

AR inhibition has profound impacts on AR protein expression, and involves complex mechanisms (Figure 6). At transcription level, ligand-activated AR binds the intron 1 of the AR gene and further recruits a corepressor complex to inhibit AR gene transcription [20]. This mechanism applies universally to AR positive prostate cancer cells, as AR inhibition increases AR-FL and AR-v7 mRNA levels in multiple cell lines (Figure S1). At the post-transcriptional level, alternative RNA splicing process is coupled with gene transcription. Splicing factors such as U2AF65 and ASF/SF2 are recruited readily to the transcribed AR pre-mRNA, resulting in rapid AR-v7 mRNA synthesis under castration conditions [12, 28]. At the post-translational level, protein kinases and phosphatases determine whether translated proteins of AR-FL and its splice variants can be stabilized to exert their functions. In LNCaP and LNCaP95 cells, MAB enhances Akt activity but reduces PP-1 expression. The net outcome is enhancement of AR pSer(213) and acceleration of AR protein degradation. In 22Rv1 cells, AR inhibition increases PP-1 expression, while Akt activity remains at minimal levels. Reduced AR pSer(213) therefore stabilizes AR-FL and AR-v7 proteins. However, in VCaP cells both PP-1 and Akt signaling are not affected by MAB. MAB increases AR-v7 expression through upregulating AR gene transcription and RNA splicing.

**Figure 6:** A summary of regulatory mechanisms that control AR-v7 protein expression

Our results indicate that AR-FL and AR-v7 share the same mechanism of Mdm2 mediated ubiquitin-proteasome degradation process. However, these studies highlight that under AR inhibition conditions where AR-FL function is potently suppressed, the protein expression of AR-v7 becomes significantly important due to its constitutively and transcriptionally active nature, and its effectiveness in driving CRPC progression. Furthermore, our results indicate that PP-1 can induce de-phosphorylation of Serine 213 of AR-v7 and AR-v7 protein stabilization, suggesting that similar PP-1 action may also apply to AR-FL. PP-1 may exert its function through either directly de-phosphorylating pSer213 of AR-v7 or indirectly through de-phosphorylating, thereby deactivating Akt. Together, these results suggest that through modulating PP-1 activity, we may control AR-v7 as well as AR-FL protein expression in prostate cancer cells.

In summary, we define the molecular mechanisms by which PP-1 and Akt signaling can regulate serine 213 phosphorylation of AR-v7, and thereby AR-v7 protein expression in cell genetic background-dependent manners. These findings provide new insights into resistant mechanisms of CRPC. They also suggest that profiling PP-1 and Akt signaling in CRPC patients would be useful to develop personalized therapeutic strategy in order to demolish AR signaling more efficiently in prostate tumors.

## MATERIALS AND METHODS

### Cell culture and transfection

LNCaP, 22Rv1, VCaP, PC3 and 293T cell lines were purchased from ATCC (Manassas, VA, USA). The LNCaP95 cell line was a generous gift from Dr. Alan Meeker of Johns Hopkins University. Cells were maintained in phenol red free RPMI1640 medium containing 5% charcoal stripped serum as we have shown [12, 29]. LNCaP and 22Rv1 cells were cultured in RPMI1640 medium, while other lines were maintained in Dulbecco's Modified Eagle Medium (DMEM). LNCaP(AR-v7), PC3(AR-v7) and PC3(AR-FL) are cell lines where AR-v7 or AR-FL are introduced by lentiviral infection and selected by blasticidin using the protocol we reported [30, 31]. Plasmid DNA transfection was performed by using Liofectamine2000 (Life Technology), while siRNAs were transfected by using siLentFect (Bio-Rad) according to the manufacturer's protocol. Detailed information on plasmid DNA, siRNA and chemicals is listed in materials. The AR-v7 mutant plasmids were generated with a site-directed mutagenesis kit (New England Biolabs).

### Real-time qPCR

Total RNA was extracted by TRIZOL reagent (Invitrogen), treated with deoxyribonuclease and reversely transcribed by random hexamers and superscript II (Invitrogen). Real-time qPCR was performed on the ABI PRISM 7900 HT system (Applied Biosystems) using the FastStart Universal SYBR Green Master mix (Roche) following standard protocol as we reported [30]. All real-time qPCR assays were carried out in triplicates from three independent cDNA syntheses. Primer information is listed in the materials.

### Immunoblotting and immunoprecipitation (IP)

Whole cell lysates were extracted by the buffer containing 50mM of Tris pH8.0, 150mM of NaCl, 1% NP40, 0.5% sodium deoxycholate, 0.1% SDS and proteinase and phosphatase inhibitors (Roche). A nuclear protein extraction kit (Sigma) was used to isolate cytoplasm and nuclear proteins according to the manufacturer's instruction. Immunoblotting assays follow the standard protocol as reported [30]. Information on antibodies is listed in materials. When performing co-IP assays, cell lysates were extracted by NETN buffer containing 0.5% NP40, 1mM of EDTA, 50mM of Tris, and 150mM of NaCl plus proteinase and phosphatase inhibitor (Roche). Pre-cleared lysates were incubated with AR or Mdm2 antibody, and the associated proteins were immunoblotted by antibodies as indicated. Experiments were repeated at least three times, and one set of the representative blots was shown. Densitometry analyses of protein bands were performed by Image J software.

### *In vivo* ubiquitination assay

An *in vivo* ubiquitination assay was carried as described previously [31] with a modification where 2% SDS was applied to induce a denature condition. Cells were transfected with plasmids encoding HA-tagged ubiquitin (3μg) and AR-FL or AR-v7 (6μg) and treated with 2μg/ml of MG132 for 16 hours. Cells were also transfected with Mdm2 plasmid (6μg), PP-1 plasmid (6μg), cAkt or dAKT plasmid (6μg) or treated with 5μM of TMC as indicated in figures. Whole cell lyses were extracted using a buffer containing 50mM of Tris pH8.0, 150mM of NaCl, 1% NP40, 0.5% sodium deoxycholate, 2% SDS and proteinase and phosphatase inhibitors (Roche). Cytosol and nuclear protein lyses were extracted using a NE-PER nuclear and cytoplasmic extraction Kit (Life Technology). Lyses were added with 2% SDS, heated at 95°C for 5 minutes, and diluted 10 times before being subjected to immunoprecipitation with the AR antibody. Precipitated proteins were then immunoblotted with both ubiquitin and AR antibodies.

### Immunofluorescence staining

Cells were fixed in 4% paraformaldehyde, permeabilized in 0.25% Triton X-100, and blocked with 1% BSA for 1 hour at room temperature. Cells were then incubated with the primary antibody, washed with PBS with 0.1% Triton X-100, and incubated with FITC-conjugated secondary antibody (1:1000 in PBST containing 1% BSA). Cell imaging was captured by a Zeiss fluorescent microscope (Carl Zeiss, Thornwood, NY).

### Luciferase reporter assay

Cells were transfected with PSA-luciferase reporter plasmid with the renilla reporter as a control for transfection efficiency. Luciferase activities were determined using the luciferin reagent (Promega, Madison, WI) according to the manufacturer's protocol. Transfection efficiency was normalized by renilla luciferase activity.

## SUPPLEMENTARY MATERIAL FIGURES AND TABLES


